# The Significance of Implementing Bilevel Positive Airway Pressure under Cluster Nursing in Improving the Survival Possibility of Patients with Severe Pulmonary Infection Complicated by Respiratory Failure

**DOI:** 10.1155/2022/2324797

**Published:** 2022-09-19

**Authors:** Xiao Fang, Haiyan Yang

**Affiliations:** Department of Emergency Intensive Care Unit, Nanjing First Hospital, Nanjing Medical University, Nanjing, Jiangsu 210014, China

## Abstract

**Objective:**

To explore the significance of bilevel positive airway pressure (BIPAP) under cluster nursing in improving the survival probability of patients with severe pulmonary infection (SPI) complicated by respiratory failure (RF).

**Methods:**

This research included 153 SPI patients complicated by RF (SPI + RF) admitted between January 2020 and March 2022, including 55 cases in group A who were treated with BIPAP under cluster care during hospitalization, 47 cases in group B receiving invasive continuous mechanical ventilation during hospitalization, and 51 cases in group C treated with BIPAP under routine care during hospitalization. The three cohorts were compared regarding pre- and posttreatment serum inflammatory factors (IFs), blood gas (BG) parameters, heart rate (HR), and respiratory rate (RR). Besides, the cumulative time of ventilator use, successful ventilator weaning rate, mortality, and incidence of adverse events were counted. Finally, patients were scored for their psychological state using the Hamilton Anxiety/Depression Scale (HAMA/HAMD).

**Results:**

The posttreatment TNF-*α*, IL-6, PCT, WBC, and PaCO_2_ reduced statistically in all the three groups, with the lowest levels found in group A and the highest in group B (*P* < 0.05); while PaO_2_ and SpO_2_ increased, with the highest values found in group A and the lowest in group B (*P* < 0.05). Among the three groups, group A had the shortest duration of ventilator use, the highest successful weaning rate, and the lowest incidence of adverse events (*P* < 0.05). Besides, HAMA and HAMD scores were the lowest in group A among the three groups, while those in group B were higher compared with group C (*P* < 0.05).

**Conclusion:**

The implementation of BIPAP under cluster nursing can effectively reduce inflammatory responses of SPI + RF patients, improve their vital signs, and enhance their psychological state, which has extremely high clinical application value.

## 1. Introduction

Pulmonary infection (PI) refers to inflammation of the lung parenchyma due to infection, usually caused by virus or bacterial infection [1]. The incidence of PI keeps increasing, in parallel with the aging of population in China [2]. In addition, due to the continuous decline of physical function in the elderly population, once pulmonary infection occurs, most of the cases are severe and difficult to treat [3]. Moreover, PI can lead to hypoxia and metabolic dysfunction, which can easily cause respiratory failure (RF) and other complications, posing a serious threat to patients' life safety [4]. Therefore, timely and effective treatment is of great clinical significance to reduce the mortality of severe pulmonary infection (SPI) complicated with RF (SPI + RF) and improve patients' outcomes [5].

The traditional treatment of SPI + RF mainly adopts tracheal intubation and ventilators [6]. Although this can establish an effective artificial respiration channel and maintain the patient's normal breathing, it is very likely to cause severe invasive stress and inflammatory reactions after intubation, resulting in other complications [7]. At the same time, endotracheal intubation will also make the patient very uncomfortable and increase the pain of the patient [8]. Not only that, but more and more studies have pointed out that the success rate of endotracheal intubation is getting lower and lower in recent years [9, 10]. In contrast, bilevel positive airway pressure (BIPAP), with the advantage lay in the noninvasive treatment that can lower the risk of traumatic infection and reduce complications and improve safety, has been well received in clinic [11]. In addition, effective nursing intervention during treatment for patients with SPI + RF has been shown to reduce complications and significantly improve the prognosis of patients after treatment [12].

The application of personalized nursing strategies in disease treatment has gradually become a clinical consensus. For example, continuous nursing based on the Omaha system can improve the fatigue and mental state of patients with lung cancer during chemotherapy [13], and nursing care given at home can improve the quality of life of patients with gastric cancer [14] and so on. This fully shows that the development of personalized nursing strategies has an important effect on improving the treatment effect of various diseases. Of them, cluster nursing, a comprehensive and continuous nursing plan integrating the practice of evidence-based hospitals and patients' conditions, has achieved excellent results in the treatment of pressure ulcers, gastroenteritis, and other diseases as well as in the intensive care unit (ICU) [15–17]. However, its employment in SPI + RF and bilevel positive airway pressure (BIPAP) remains rarely reported.

We speculate that cluster nursing can effectively improve the patient's treatment experience and safety during the BIPAP treatment of patients with SPI combined with RF, which is of great significance to the patient's rehabilitation. Consequently, this research is carried out to provide effective treatment measures for the future clinical treatment of SPI + RF and reduce its harm.

## 2. Materials and Methods

### 2.1. Study Area

The study was carried out at department of emergency intensive care unit, Nanjing First Hospital from January 2020 to April 2022.

### 2.2. General Information

This research enrolled 153 SPI + RF patients admitted between January 2020 and March 2022 and grouped them as follows based on the difference in the treatment and care during hospitalization: group A (*n* = 55; BIPAP under cluster care), group B (*n* = 47; invasive continuous mechanical ventilation), and group C (*n* = 51; BIPAP under routine care). This study was conducted in strict accordance with the Declaration of Helsinki, and all subjects in the study signed the informed consent form by the patients themselves (or their immediate family members).

### 2.3. Eligibility Criteria

The included participants were all diagnosed as SPI by X-ray examination, arterial blood analysis, and routine blood tests and met the diagnostic criteria for RF [18] and all indications for mechanical ventilation [19], with complete medical records and no serious medical diseases nor lung tumors. On the contrary, those with severe liver and kidney dysfunction, mental disorders, RF caused by other diseases, drug allergies, or immune diseases were excluded. Besides, referrals, as well as those who refused, contradicted medical investigators and were unable to take care of themselves were ruled out.

### 2.4. Treatment Schemes

After admission, all patients were given routine treatments such as anti-inflammatory, blood pressure maintenance, cough relief, expectorant, and water-electrolyte balance adjustment. BIPAP: a Philips Respironics bilevel ventilator was adopted, and the nasal mask was selected, which was adjusted to self-trigger time control mode. The initial value was set to 6-8 cm H2O, which was gradually increased to an appropriate level within 5-20 minutes; the positive expiratory pressure was 4-6 cm H2O and could be increased according to the patient's RF degree. In patients with spontaneous breathing, the inspiratory time was usually set as 0.8-1.2 s with the inspiratory ratio of 1 : 1.5-2.0. At the beginning of ventilation, the nursing staff paid close attention to the patient's flatulence and other adverse reactions to make timely adjustments. In addition, according to the specific situation of the patient, the ventilator was temporarily stopped to perform operations such as drinking water and expectorating sputum, and weaning was performed until the patient could complete spontaneous breathing. Invasive continuous mechanical ventilation: first, an artificial airway was established, and the auxiliary control ventilation mode was used. When the patient's spontaneous breathing frequency was lower than the preset frequency or the patient's inspiratory efforts cannot trigger the ventilator, BIPAP was performed with the preset tidal volume and ventilation frequency; and if the patient's inspiratory can trigger the ventilator, the ventilation was performed with a higher frequency than the preset frequency and then gradually transition to synchronous intermittent mandatory pressure support ventilation until weaning.

### 2.5. Nursing Measures

Routine nursing: nursing staff informed patients of the treatment principles, precautions, and other contents, so that patients can better cooperate to complete the treatment. Basic psychological counseling was also given to eliminate patients' adverse emotions. The ward was maintained quiet and clean to create a good environment. Besides, patients' vital signs were closely watched, the respiratory tract was kept unobstructed, and sputum aspiration was provided. Cluster nursing: nursing staff involved in cluster nursing all mastered certain professional knowledge. A working group was established to discuss and improve nursing contents and implement nursing intervention strictly according to the plan. In addition, nurses took the initiative to communicate with patients to share past successful cases, as well as disease-related knowledge, matters needing attention in daily life, so as to improve patients' confidence in treatment and degree of coordination. Family members were also instructed to understand and master the relevant dietary management, so that patients eat high protein and vitamin foods. Furthermore, the respiratory tract care of the patients was carried out by special personnel, and sputum suction machines were used if necessary for those with cough difficulties. Moreover, oral care was given regularly, and medical instruments and ventilator pipes were disinfected regularly. After weaning, patients were assisted to complete simple rehabilitation training, the oxygen demand was ensured, and their vital signs were closely observed.

### 2.6. Endpoints

Serum inflammatory factors (IFs), including tumor necrosis factor *α* (TNF-*α*), interleukin 6 (IL-6), procalcitonin (PCT), and white blood cell (WBC), were detected by ELISA before and after treatment. A blood gas (BG) analyzer detected the following BG parameters before and after treatment: oxygen partial pressure (PaO_2_), arterial partial pressure of carbon dioxide (PaCO_2_), and blood oxygen saturation (SpO_2_). Pre- and posttreatment heart rate (HR) and respiratory rate (RR) were also recorded. The cumulative time of ventilator use, successful weaning rate (number of people who successfully removed mechanical ventilation equipment/total number × 100%), mortality (patients who died during treatment/total number × 100%), and incidence of adverse reactions (the number of adverse reactions/total number × 100%) were counted. Hamilton Anxiety Scale (HAMA) and Depression Scale (HAMD) were utilized for psychological state evaluation of patients [20]: the HAMA score includes 14 items, and the HAMD score includes 17 items. The alternative answers are asymptomatic, mild, moderate, severe, and very severe, with scores ranging from 0 to 4, with higher scores representing anxiety (depression) the more serious the situation is.

### 2.7. Statistics and Methods

SPSS23.0 performed statistical analysis of the data. The Chi-square test identified the differences of count data denoted by (%); one-way ANOVA and LSD intragroup tests were used for comparison of measurement data expressed as (^−^*χ* ± *s*). Statistical significance was indicated by *P* < 0.05.

## 3. Results

### 3.1. Summary of Results

In this experiment, the posttreatment TNF-*α*, IL-6, PCT, WBC, and PaCO2 reduced statistically in all the three groups, with the lowest levels found in group A and the highest in group B (*P* < 0.05); while PaO2 and SpO2 increased, with the highest values found in group A and the lowest in group B (*P* < 0.05). Among the three groups, group A had the shortest duration of ventilator use, the highest successful weaning rate, and the lowest incidence of adverse events (*P* < 0.05). Besides, HAMA and HAMD scores were the lowest in group A among the three groups (*P* < 0.05).

### 3.2. Patient Data

Patients' clinical data like age, BMI, sex, living environment, disease type, ethnicity, and smoking history were collected and statistically analyzed (Table 1). The results showed that there were no significant differences in age, BMI, gender, living environment, disease type, ethnicity, and smoking history among the three groups (*P* > 0.05), confirming that the three groups were comparable.

### 3.3. Alterations of Pre- and Posttreatment IFs

First, we detected pre- and posttreatment alterations in IFs in the three groups. The results identified nonsignificant differences among the groups prior to treatment (*P* > 0.05) and notably reduced levels after treatment (*P* < 0.05). The posttreatment TNF-*α* levels in groups A, B, and C were (2.48 ± 0.21) mg/L, (3.14 ± 0.33) mg/L, and (2.93 ± 0.25) mg/L, respectively, with the lowest in group A and the highest in group B (*P* < 0.05, Figure 1(a)). The posttreatment IL-6 levels in groups A, B, and C were (8.44 ± 0.78) *μ*g/L, (11.07 ± 1.10) *μ*g/L, and (9.65 ± 0.66) *μ*g/L, respectively, with the level in group C higher than group A and lower than group B (*P* < 0.05, Figure 1(b)). The comparison of posttreatment PCT levels among the three groups also revealed the lowest level in group A and the highest in group B (*P* < 0.05, Figure 1(c)). At last, the WBC of group A after treatment was (10.46 ± 2.87) × 109/L, which was lower compared with groups B and C; the WBC of group B after treatment was (14.86 ± 3.08) × 109/L, higher versus group C (*P* < 0.05, Figure 1(d)).

### 3.4. Alterations of Pre- and Posttreatment BG Function

Subsequently, we compared alterations in BG function among the three groups. The results also determined no difference in pretreatment PaO_2_, PaCO_2_, and SpO_2_ among the three groups (*P* > 0.05). Increased PaO_2_ was observed in all the three groups after treatment, with the highest and the lowest level found in group A (71.91 ± 6.60 mmHg) and group B (59.92 ± 6.47 mmHg), respectively (*P* < 0.05, Figure 2(a)). A decrease in PaCO_2_ was found in all the three groups after treatment; the posttreatment PaCO_2_ in group A was (37.28 ± 3.70) mmHg, which was lower versus groups B and C, while that in group B was (44.98 ± 4.61) mmHg, higher than group C (*P* < 0.05, Figure 2(b)). SpO_2_ was also elevated in the three groups after treatment, and the increase in Group A was the most significant, followed by group C (*P* < 0.05, Figure 2(c)).

### 3.5. Changes in Pre- and Posttreatment Vital Signs

Similarly, HR and RR differed insignificantly among the three groups prior to treatment (*P* > 0.05). After treatment, the HR of group A was (80.47 ± 4.90) beats/min, which was lower versus groups B and C, while the HR of group B was (92.06 ± 5.15) beats/min, higher than that of group C (*P* < 0.05, Figure 3(a)). The posttreatment RR levels of groups A, B, and C were (20.8 ± 22.04) times/min, (25.02 ± 1.85) times/min, and (22.65 ± 0.06) times/min, respectively, with that in group A being the highest and that in group B higher than group C (*P* < 0.05, Figure 3(b)). The posttreatment HR and RR in both groups was decreased compared with their pretreatment levels (*P* < 0.05).

### 3.6. Comparison of Therapeutic Effects

All patients in groups A and C were treated successfully with no patient death, while one patient died in group B. The three groups presented no significant difference in mortality (*P* > 0.05). The duration of ventilator use in groups A, B, and C was (95.08 ± 16.31) h, (114.25 ± 25.66) h, and (101.62 ± 15.10) h, respectively, with that in group B being the longest and that in group A being the shortest (*P* < 0.05). In addition, the successful weaning rate of group A was 100%, versus 98.04% in group C, with no marked difference between them (*P* > 0.05); while the successful weaning rate of group B was only 91.49%, lower than that of group A (*P* < 0.05, Table 2).

### 3.7. Comparison of Incidence of Adverse Reactions

Over the course of treatment, the incidence of adverse events observed in group A was 5.45%, the lowest of the three groups (*P* < 0.05); the incidence in group B was 29.79%, which was not significantly different from 13.73% in group C (*P* < 0.05), but higher than Group A (*P* < 0.05, Table 3).

### 3.8. Comparison of Psychological Scores

Finally, we evaluated and compared patients' psychological status among the three groups. HAMA and HAMD scores in group A were calculated to be (22.55 ± 1.92) and (24.78 ± 1.69), respectively, which were the lowest among the three groups. While HAMA and HAMD scores in group B were (34.30 ± 1.76) and (34.98 ± 2.07), respectively, which were higher versus group A. HAMA and HAMD scores in group C were higher compared with group A and lower versus group B (*P* < 0.05, Figures 4(a) and 4(b)).

## 4. Discussion

At present, the treatment of SPI patients mainly focuses on anti-infection, maintenance of patients' respiratory function, and improvement of acid-base metabolism balance [21, 22]. Among them, BIPAP has gradually become the first choice for SPI + RF, and how to further improve the therapeutic efficacy of patients is the hotspot of clinical research [23–25]. Therefore, this study may be of great implications for the application of BIPAP under cluster nursing and for further improving the therapeutic effect of SPI + RF in the future.

Endotoxin produced by pathogens can stimulate immune cells to release massive inflammatory factors, leading to endothelial cell adhesion and neutrophil proliferation, during which proteases are released in large quantities, causing damage to vascular endothelial cells and epithelial cells, and finally causing pulmonary fibrosis and microthrombosis [26, 27]. Therefore, the level of IFs in the body is of great significance in evaluating the development of SPI + RF. In this research, TNF-*α*, IL-6, PCT, and WBC were reduced statistically in all the three groups after treatment, with lower levels in groups A and C compared with group B, indicating that BIPAP was better than conventional mechanical ventilation in alleviating patients' inflammatory responses, which was consistent with past literature [28, 29]. Besides, we found better improved BG function and vital signs in groups A and C after treatment, further demonstrating the excellent application effect of BIPAP. Previous studies have suggested that BIPAP therapy can warm and humidify the inhaled gas through the upper respiratory tract, meet the needs of mask mechanical ventilation, shorten the hospitalization time of RF patients, and reduce the rate of tracheal intubation; in SPI, it can also effectively remove a large amount of inflammatory secretions in the airway, reduce airway obstruction, and improve lung ventilation and ventilation function [30, 31]. Therefore, under BIPAP, not only the high resistance in the airway can be overcome but also the workload of the respiratory muscles and the oxygen consumption can be reduced, so as to avoid the overwork of the respiratory muscles, improve the compliance of the lungs, and adjust the oxygen partial pressure, ultimately lowering the possibility of damage to the body and other organs. This study identified a lower incidence of adverse reactions in groups A and C compared with group B, which can also illustrate this point of view. Second, better survey results and lower HAMA and HAMD scores were determined in group A versus group C, which we think is due to the application effect of cluster nursing. Through cluster nursing, the professionalism and dynamics of nursing services can be guaranteed, reflecting the pertinence and integrity of nursing measures [32, 33]. Among them, the psychological attention to patients can enable them to fully understand the treatment methods and related operations, as well as self-regulation of bad emotions. Postural care can prevent reflux, aspiration, etc., to improve the comfort of treatment. Phlegm-expelling nursing is the focus of cluster nursing, which aims to ensure the unobstructed respiratory tract. Diet care can scientifically guide patients' diet and ensure balanced nutrition. And regular cleaning of oral secretions in oral care can ensure oral hygiene and avoid complications such as flatulence. All these measures of cluster nursing explain significantly accelerated physical rehabilitation and psychological improvement of patients compared with conventional nursing, indicating the important role of cluster nursing in future treatment of SPI + RF. In a previous study, we also found that cluster nursing can also reduce bilirubin levels, improve jaundice symptoms, and shorten the course of the disease in neonatal ABO solution treatment [34]; this also illustrates once again the citation value of cluster nursing in clinical practice. And for patients with gestational hypertension combined with osteoarthritis, the use of cluster nursing can reduce patient negative emotions, increase satisfaction, and improve maternal and infant outcomes [35]. It can be seen that cluster nursing is suitable for patients with various diseases, different genders, and different ages and has important clinical research significance.

Of course, due to the small number of cases included in this experiment, there may be chance of statistical calculation results, so we need to include more patient data for verification in the follow-up. Second, since there is no unified guideline for cluster nursing in clinic at present, the specific protocols implemented in this study may still have room for improvement. In addition, we need to follow up all study subjects for a longer time to evaluate their long-term outcomes.

## 5. Conclusion

The implementation of BIPAP under cluster nursing can effectively reduce inflammatory responses of SPI + RF patients, improve their vital signs, and enhance their psychological state, which has extremely high clinical application value.

## Figures and Tables

**Figure 1:** Alterations of pre- and posttreatment IFs. (a) Comparison of TNF-*α* among the three groups before and after treatment. (b) Comparison of IL-6 among the three groups before and after treatment. (c) Comparison of PCT among the three groups before and after treatment. (d) Comparison of WBC among the three groups before and after treatment. ^∗^*P* < 0.05 compared to before treatment, ^&^*P* < 0.05 compared to group A, ^#^*P* compared to group B.

**Figure 2:** Alterations of pre- and posttreatment BG function. (a) Comparison of PaO2 among the three groups before and after treatment. (b) Comparison of PaCO2 among the three groups before and after treatment. (c) Comparison of SpO2 among the three groups before and after treatment. ^∗^*P* < 0.05 compared to before treatment, ^&^*P* < 0.05 compared to group A, ^#^*P* compared to group B.

**Figure 3:** Changes in pre- and posttreatment vital signs. (a) Comparison of HR among the three groups before and after treatment. (b) Comparison of RR among the three groups before and after treatment. ^∗^*P* < 0.05 compared to before treatment, ^&^*P* < 0.05 compared to group A, ^#^*P* compared to group B.

**Figure 4:** Comparison of psychological scores. (a) Comparison of HAMA scores. (b) Comparison of HAMD Scores. ^∗^*P* < 0.05 compared to group A, ^#^*P* compared to group B.

**Table 1:** Patient data.

	Group A (*n* = 55)	Group B (*n* = 47)	Group C (*n* = 51)	*F* or *χ*^2^	*P*
Age	64.6 ± 5.5	65.6 ± 4.1	64.9 ± 3.9	0.621	0.539
BMI (kg/m^2^)	25.61 ± 4.27	26.50 ± 3.36	26.02 ± 3.54	0.707	0.495
Gender				0.020	0.990
Men	32 (58.18)	28 (59.57)	30 (58.82)		
Woman	23 (41.81)	19 (40.23)	21 (41.18)		
Type of disease				0.136	0.998
Infectious pneumonia	30 (54.55)	26 (55.32)	29 (56.86)		
Aspiration pneumonia	17 (30.91)	15 (31.91)	15 (29.41)		
Bronchiolitis	8 (14.51)	6 (12.77)	7 (13.73)		
Nationality				1.024	0.599
Han	50 (90.91)	45 (95.74)	48 (94.12)		
Minority	5 (9.09)	2 (4.26)	3 (5.88)		

**Table 2:** Comparison of therapeutic effects.

	Group A (*n* = 55)	Group B (*n* = 47)	Group C (*n* = 51)	*F* or *χ*^2^	*P*
Time of ventilator use (h)	95.08 ± 16.31	114.25 ± 25.66^∗^	101.62 ± 15.10^∗^^#^	12.700	<0.001
Successful weaning rate	55 (100.0)	43 (91.49%)^∗^	50 (98.04)	6.220	0.045
Mortality	0 (0.0)	1 (2.13%)	0 (0.0)	2.270	0.321

**Table 3:** Comparison of incidence of adverse reactions.

	Group A (*n* = 55)	Group B (*n* = 47)	Group C (*n* = 51)	*χ* ^2^	*P*
Bloating	1 (1.82)	4 (8.51)	2 (3.92)		
Sore throat	1 (1.82)	5 (10.64)	2 (3.92)		
Malnutrition	0 (0.0)	2 (4.26)	1 (1.96)		
Chest tightness	1 (1.82)	3 (6.38)	2 (3.92)		
Incidence of adverse reactions (%)	5.45%	29.79%^∗^	13.73%	11.570	0.003

## Data Availability

The datasets used and/or analyzed during the current study are available from the corresponding author on reasonable request.
